This article has been retracted.

# Spontaneous Rupture of Large Angiomyolipoma of the Kidney: A Rare Case

**DOI:** 10.7759/cureus.19908

**Published:** 2021-11-25

**Authors:** Rakan M Altuwayr, Fahad S Almutairi, Shuruq H Alkhaibari, Abdullah M Alharbi, Abdullah A Alramih, Raghdah A Alamri, Alwaleed S Alghamdi, Mishari M Alshammari, Thurya S Alshammari, Abdulmajeed A Alzahrani, Dina M Al Khafaji, Abdulrahman A Alamri, Khalid A Alshahrani, Sara A Binsalman, Faisal Al-Hawaj

**Affiliations:** 1 College of Medicine, Vision Colleges, Riyadh, SAU; 2 College of Medicine, Taif University, Taif, SAU; 3 College of Medicine, Qassim University, Buraydah, SAU; 4 College of Medicine, Dar Al Uloom University, Riyadh, SAU; 5 College of Medicine, Imam Abdulrahman Bin Faisal University, Dammam, SAU; 6 College of Medicine, King Abdulaziz University, Jeddah, SAU; 7 College of Medicine, Majmaah University, Al Majma'ah, SAU; 8 College of Medicine, University of Hail, Hail, SAU; 9 College of Medicine, Northern Border University, Arar, SAU; 10 College of Medicine, Dammam University, Dammam, SAU; 11 College of Medicine, King Khalid University, Abha, SAU; 12 College of Medicine, Ibn Sina National College For Medical Studies, Jeddah, SAU

**Keywords:** case report, flank pain, hemorrhage, renal angiomyolipoma, wunderlich syndrome

## Abstract

Angiomyolipoma is the most frequent neoplasm of the kidney. It may have a wide range of clinical manifestations, but it is usually detected incidentally on cross-sectional images. Rupture and hemorrhage of angiomyolipoma is an important concern for large lesions. We present the case of a 42-year-old female, with no history of urinary stones, who presented with a sudden-onset left flank pain for eight hours. Upon examination, she was tachycardic and hypotensive. Abdominal examination revealed a left-sided flank mass. Abdominal computed tomography (CT) scan with intravenous contrast demonstrated a heterogeneous mass lesion in the left kidney with mixed attenuation and had a macroscopic fat density that was surrounded by a large hematoma. Subsequently, transcatheter renal artery embolization was performed with no complications. The procedure was able to control the active bleeding. Then, a total nephrectomy was performed, and the hematoma was evacuated during laparotomy. Spontaneous nontraumatic renal hemorrhage is a very rare condition. Clinicians should keep a high index of suspicion for this condition when they encounter a patient with the clinical triad of flank pain, flank mass, and hypotension. The case demonstrated the role of endovascular embolization of angiomyolipoma to control life-threatening hemorrhage.

## Introduction

Angiomyolipoma is the most common benign solid tumor of the kidney. It has female predilection and is often identified in adulthood [1]. This tumor is composed of three components: blood vessels, spindle cells, and adipose tissues. In the majority of cases, the tumor occurs sporadically. Most cases of angiomyolipoma are detected incidentally by cross-sectional images [2]. However, renal angiomyolipoma can present with a wide range of signs and symptoms, including flank mass, hematuria, urinary tract infection, hypertension, and renal failure. Despite its benign behavior, the risk of spontaneous rupture and bleeding is a major concern of angiomyolipoma [3]. Here, we present the case of a middle-aged woman with spontaneous rupture of undiagnosed angiomyolipoma that was managed by endovascular embolization and subsequent surgery.

## Case presentation

We present the case of a 42-year-old female who was brought to the emergency department by ambulance because she developed a sudden-onset left flank pain for eight hours before presentation. The pain was non-radiating, and she described it as stabbing in nature. It was associated with nausea and dizziness. She scored the pain as 8 out of 10 on the severity scale. She reported that the pain was not related to urination, posture, or meals. The patient used over-the-counter analgesics for the pain with no clinical improvement. The medical history of the patient was remarkable for beta-thalassemia minor and allergic rhinitis. She underwent a tonsillectomy at the age of 14 years. She was not on any medications. The patient reported having an allergy to penicillin. She was a nonsmoker and never consumed alcohol. The family history was significant for glucose-6-phosphate dehydrogenase deficiency.

Upon examination, the patient was in severe pain and appeared pale and sweaty. She did not have any signs of respiratory distress. Her vital signs included tachycardia (120 bpm), hypotension (88/50 mmHg), normal respiratory rate (14 bpm), and normal temperature (36.8°C). Abdominal examination revealed a left-sided mass with generalized tenderness. Considering the hypovolemic status of the patient, aggressive intravenous hydration was initiated.

The initial laboratory investigations revealed a decreased hemoglobin level (10.9 g/dL) with normal leukocytes (8,500/μL) and platelets (380,000/μL). She also had a mild elevation in the urea and creatinine levels. Urinalysis findings were normal. The liver function test and inflammatory markers were within the reference range (Table 1).

**Table 1:** Summary of the results of the laboratory findings

Laboratory Investigation	Unit	Result	Reference Range
Hemoglobin	g/dL	10.9	13.0–18.0
White Blood Cell	1000/mL	8.5	4.0–11.0
Platelet	1000/mL	380	140–450
Erythrocyte Sedimentation Rate	mm/hour	12	0–20
C-Reactive Protein	mg/dL	3.5	0.3–10.0
Total Bilirubin	mg/dL	0.8	0.2–1.2
Albumin	g/dL	3.9	3.4–5.0
Alkaline Phosphatase	U/L	51	46–116
Gamma-Glutamyltransferase	U/L	18	15–85
Alanine Transferase	U/L	16	14–63
Aspartate Transferase	U/L	20	15–37
Blood Urea Nitrogen	mg/dL	18	7–18
Creatinine	mg/dL	1.0	0.7–1.3
Sodium	mEq/L	136	136–145
Potassium	mEq/L	3.9	3.5–5.1
Chloride	mEq/L	104	98–107

After resuscitation and maintaining hemodynamic stability, the patient underwent an abdominal computed tomography (CT) scan with intravenous contrast. The scan demonstrated a heterogeneous mass lesion in the left kidney with mixed attenuation and had macroscopic fat density. The kidney was surrounded by a hematoma that exerted mass effect upon the kidney. Such findings conferred the diagnosis of ruptured renal angiomyolipoma with active hemorrhage (Figure 1).

**Figure 1:** Coronal (A) and axial (B) CT images demonstrating a large renal mass (arrow) surrounded by hematoma with evidence of active bleeding (encircled) CT: computed tomography

The case was discussed with the interventional radiology department, and the plan for embolization was made. Transcatheter renal artery angiography demonstrated abnormal vasculature. Particulate embolic agents were administered selectively to occlude the abnormal vessels (Figure 2). The embolization process was successful, and the patient developed no complications. Following the procedure, the patient was hemodynamically stable with no evidence of active bleeding.

**Figure 2:** Transcatheter renal artery angiography demonstrating the abnormal vasculature in the arterial territory with multiple aneurysms

Subsequently, a laparotomy operation was performed to resect the tumor. A total nephrectomy was performed, and the hematoma was evacuated. Histopathological examination of the specimen confirmed the diagnosis of angiomyolipoma. The patient was discharged on the fifth postoperative day. After three months of follow-up, the patient remained asymptomatic with normal renal function tests.

## Discussion

We presented the case of a middle-aged woman with angiomyolipoma that presented with spontaneous nontraumatic rupture for which she underwent endovascular embolization and surgical resection. The spontaneous nontraumatic renal hemorrhage, also known as Wunderlich syndrome, is a rare condition with bleeding in the subcapsular and perinephric spaces [4]. Wunderlich syndrome was named after the physician Carl Wunderlich who described the first case of the syndrome in 1856 [5].

Wunderlich syndrome presents with the classic triad of acute flank pain, flank mass, and signs of hypovolemic shock. As in the present case, the most common etiology of Wunderlich syndrome is a neoplastic lesion, with angiomyolipoma being the commonest [6]. In contrast, the nonneoplastic causes of Wunderlich syndrome include vascular causes such as vasculitis, arteriovenous malformation, renal vein thrombosis, and renal artery aneurysm. Further, cystic renal diseases, coagulopathy, and stone disease are also important causative factors of Wunderlich syndrome [7].

Imaging studies are crucial to making the diagnosis of Wunderlich syndrome. A computed tomography scan demonstrates the presence of hemorrhage surrounding the kidney along with the primary lesion if present. Notably, the computed tomography scan can make the diagnosis of angiomyolipoma, the most common neoplastic cause of Wunderlich syndrome, with high accuracy and confidence [8]. The management of Wunderlich syndrome depends on the overall condition of the patient. Small hemorrhage can be managed conservatively with fluid resuscitation, while interventional procedures need to be performed for large hemorrhage. In the present case, since the computed tomography scan showed evidence of active bleeding, the patient underwent endovascular embolization to stop the bleeding, and the patient underwent nephrectomy subsequently [6]. Tomita et al. [9] conducted a retrospective study involving patients who underwent transcatheter arterial embolization for renal angiomyolipoma and found that the procedure was successful in tumor shrinkage with minimal adverse effects. We proceeded with nephrectomy considering the large hematoma and tumor size [8].

## Conclusions

Spontaneous nontraumatic renal hemorrhage is a very rare condition. Clinicians should keep a high index of suspicion for this condition when they encounter a patient with the clinical triad of flank pain, flank mass, and hypotension. A computed tomography scan can make the diagnosis promptly. The case highlights the value of endovascular embolization of angiomyolipoma to control life-threatening bleeding.
